This article has been retracted.

# Adherence towards COVID-19 mitigation measures and its associated factors among Gondar City residents: A community-based cross-sectional study in Northwest Ethiopia

**DOI:** 10.1371/journal.pone.0244265

**Published:** 2020-12-30

**Authors:** Zelalem Nigussie Azene, Mehari Woldemariam Merid, Atalay Goshu Muluneh, Demiss Mulatu Geberu, Getahun Molla Kassa, Melaku Kindie Yenit, Sewbesew Yitayih Tilahun, Kassahun Alemu Gelaye, Habtamu Sewunet Mekonnen, Abere Woretaw Azagew, Chalachew Adugna Wubneh, Getaneh Mulualem Belay, Nega Tezera Asmamaw, Chilot Desta Agegnehu, Telake Azale, Animut Tagele Tamiru, Bayew Kelkay Rade, Eden Bishaw Taye, Asefa Adimasu Taddese, Zewudu Andualem, Henok Dagne, Kiros Terefe Gashaye, Gebisa Guyasa Kabito, Tesfaye Hambisa Mekonnen, Sintayehu Daba, Jember Azanaw, Tsegaye Adane, Mekuriaw Alemayeyu

**Affiliations:** 1 Department of Women’s and Family Health, School of Midwifery, College of Medicine and Health Sciences, University of Gondar, Gondar, Ethiopia; 2 Department of Epidemiology and Biostatistics, Institute of Public Health, College of Medicine and Health Sciences, University of Gondar, Gondar, Ethiopia; 3 Department of Health Systems and Policy, University of Gondar, Gondar, Ethiopia; 4 Department of Psychiatry, College of Medicine and Health Sciences, University of Gondar, Gondar, Ethiopia; 5 Department of Medical Nursing, School of Nursing, College of Medicine and Health Sciences, University of Gondar, Gondar, Ethiopia; 6 Department of Pediatric and Child Health Nursing, School of Nursing, College of Medicine and Health Sciences, University of Gondar, Gondar, Ethiopia; 7 School of Nursing, College of Medicine and Health Sciences and Comprehensive Specialized Hospital, University of Gondar, Gondar, Ethiopia; 8 Department of Health Education and Behavioral Sciences, Institute of Public Health, College of Medicine and Health Sciences, University of Gondar, Gondar, Ethiopia; 9 Department of General Midwifery, School of Midwifery, College of Medicine and Health Sciences, University of Gondar, Gondar, Ethiopia; 10 Department of Clinical Midwifery, School of Midwifery, College of Medicine and Health Sciences, University of Gondar, Gondar, Ethiopia; 11 Department of Environmental and Occupational Health and Safety Institute of Public Health, College of Medicine and Health Sciences, University of Gondar, Gondar, Ethiopia; 12 Department of Gynecology and Obstetrics, University of Gondar College of Medicine and Health Sciences, Gondar, Ethiopia; National Institute for Infectious Diseases Lazzaro Spallanzani-IRCCS, ITALY

## Abstract

**Background:**

Considering its pandemicity and absence of effective treatment, authorities across the globe have designed various mitigation strategies to combat the spread of COVID-19. Although adherence towards preventive measures is the only means to tackle the virus, reluctance to do so has been reported to be a major problem everywhere. Thus, this study aimed to assess the community’s adherence towards COVID-19 mitigation strategies and its associated factors among Gondar City residents, Northwest Ethiopia.

**Methods:**

A community-based cross-sectional study was employed among 635 respondents from April 20–27, 2020. Cluster sampling technique was used to select the study participants. Data were collected using an interviewer-administered structured questionnaire. Epi-Data version 4.6 and STATA version 14 were used for data entry and analysis, respectively. Binary logistic regressions (Bivariable and multivariable) were performed to identify statistically significant variables. Adjusted odds ratio with 95% CI was used to declare statistically significant variables on the basis of p < 0.05 in the multivariable logistic regression model.

**Results:**

The overall prevalence of good adherence towards COVID-19 mitigation measures was 51.04% (95%CI: 47.11, 54.96). Female respondents [AOR: 2.39; 95%CI (1.66, 3.45)], receiving adequate information about COVID-19 [AOR: 1.58; 95%CI (1.03, 2.43)], and favorable attitude towards COVID-19 preventive measures were significantly associated with good adherence towards COVID-19 mitigation measures. Whereas, those respondents who had high risk perception of COVID-19 were less likely to adhere towards COVID-19 mitigation measures [AOR: 0.61; 95% CI (0.41, 0.92)].

**Conclusions:**

The findings have indicated that nearly half of the study participants had poor adherence towards COVID-19 mitigation measures. Sex, level of information exposure, attitude towards COVID-19 preventive measures, and risk perception of COVID-19 were factors which significantly influenced the adherence of the community towards COVID-19 mitigation measures. Therefore, it is crucial to track adherence responses towards the COVID-19 preventive measures, scale up the community’s awareness of COVID-19 prevention and mitigation strategies through appropriate information outlets, mainstream media, and rely on updating information from TV, radio, and health care workers about COVID-19.

## Background

Coronaviruses (Cov) are a large family of viruses that cause a wide range of illnesses ranging from common cold to severe diseases [1, 2]. A novel coronavirus (nCov), also called SARS-CoV-2, is the new strain of the virus that causes respiratory illness such as common cold, Severe Acute Respiratory Syndrome (SARS) and Middle East Respiratory Syndrome (MERS) and has not been previously identified in human population [3]. The first case of the COVID-19 epidemic was discovered in Wuhan city, Hubei province of China with unexplained pneumonia on December 12, 2019, and 27 viral pneumonia cases, seven of them being severe, were officially announced on December 31, 2019 [4].

Corona virus disease 2019 (Covid-19) typically shows flu-like symptoms such as fever, loss of taste, and cough [5–7]. Though there is still much to discover about symptoms of the disease, it starts with a fever, followed by a dry cough, and it later leads to shortness of breath and sore throat. The first report from China indicated that 80% of infections are mild, and only 20% of patients (15% severe and 5% critical) require hospital admission [5, 8, 9]. COVID-19 is a new disease that is distinct from other diseases that have known so far across the globe such as SARS, MERS, and influenza. Although coronavirus and influenza infections cause similar symptoms, the new coronavirus is different with respect to significant community spread and severity [1, 10]. Globally, the virus has affected 213 countries and territories and has resulted in greater loss of life and the broader economic crisis. As of August 2, 2020, more than 18 million people have been infected and half a million deaths were caused by the pandemic worldwide [3, 11].

Considering its pandemicity and absence of effective treatment, the World Health Organization(WHO) has designed various mitigation strategies to combat the spread of COVID-19. Among these, staying at home, social distancing, wearing masks, and applying hand hygiene are the common precaution measures to break the pandemic. In addition, in response to the pandemic, countries across the globe have taken various measures to slow the spread of the virus down and protect vulnerable groups from getting infected of the virus [12]. These measures are vital in decreasing mortality and reducing the overburden of the health care systems [13, 14]. Such protective measures are believed to decrease further COVID-19 transmissions overall and in particular to protect individuals at increased risk for severe illness including older adults, people with underlying medical conditions, and frontline health workers in particular [15–17].

Despite the repeated consensus that adhering towards such guidelines is the most effective way to defuse the novel coronavirus, community’s risk perception and poor adherence towards COVID-19 mitigation measuresremain problems. A significant proportion of communities did not perceive the virus as a risk for health. People also think that it originated from a laboratory, and mostly causes mild symptoms, and affects the elderly [18, 19]. These negative behaviors toward COVID-19 in the community across the world remain a great concern and can be mainly associated with lack of knowledge, misperception about the disease [15], lack of appropriate information, and the social and economic factors as well as lack of government concern. Although people’s adherence towards mitigation measures is highly affected by their knowledge, behavior and practices, a lot of information they get in this area might be fake and infodemic that potentially disturb the public and influence their measures [15, 20]. Furthermore, most people supposed that COVID-19 is a stigmatized disease despite efforts on risk communication and public education [20, 21].

In Ethiopia, there is an increasing number of COVID-19 cases. As of August 2, 2020, a total of 17,999 confirmed cases and 284 deaths are reported. By August 6th, Ethiopia had recorded 20,900 cases and 365 deaths, with a recent upsurge since mid-July, particularly in the last fortnight. One-fifth of the cases (20%) but more than a quarter of the deaths (28%) occurred in the past seven days, suggesting that the rate of mortality and the number of critical cases is increasing. Ethiopia ranks 68th worldwide and 8th in Africa with South Africa in the lead followed by the two other countries with a population of more than 100 million: Egypt and Nigeria, which have much lower numbers tested overall and per million inhabitants than Ethiopia [22].

Since COVID-19 has been declared as a public health threat globally and nationally, the Ethiopian government initiated a screening program, established quarantine and treatment centers in addition to community awareness and strong enforcement to slow the nationwide spread of the virus. In Gondar city, where the study was conducted, the risk of COVID-19 has become high. The closeness of the city to the Sudanese border and the city’s tourist destinations will make it the second epicenter next to Addis Ababa. To this effect, there is a need for information about the community’s adherence towards the recommended mitigationmeasures. However, to date, there is no study that assessed community’s adherence towards COVID-19 pandemic in the study area. Therefore, our study aimed to assess the community’s adherence towards COVID-19 mitigation strategies and its associated factors among residents of the city of Gondar, Northwest Ethiopia. The findings of this study will help local decision makers and COVID-19 task forces to design an effective intervention against the pandemic.

## Methods

### Study area

The study was conducted in Gondar city, Amhara regional state, Northwest Ethiopia. The city is located in Central Gondar Zone, Amhara Regional State, and is 748 km far from Northwest of Addis Ababa, the capital of Ethiopia and, about 180 kilometers from Bahir Dar city, the capital of Amhara regional state. It has an altitude of 12°36′N 37°28′E and longitude of 12.60N 37.467’E with an elevation of 2133 meters above sea level and is divided into 12 administrative areas (sub-cities) which consist of 21 kebeles (the smallest administrative units in Ethiopia). Gondar is among one of the ancient and largely populated cities in the country. The city has now one comprehensive specialized hospital and eight health centers providing health services to the population.

### Study design and period

A community-based cross-sectional study was conducted from April 20 to 27, 2020.

### Participants

The source population were all people 18 years of age and above residing in Gondar city, while the study population were all people 18 years of age and above in the selected kebeles (the smallest administrative unit) of the city.

### Sample size calculation and sampling procedures

The sample size was determined by using single population proportion formula by considering the following statistical assumptions:

Confidence level (Cl), 95%

Proportion = 50%

Margin of error 5%

Using the following single proportion formula: -

$$n=\frac{\left(Za∕2)2\;x\;P(1-P\right)}{(W)2}$$

Where

n = initial sample size

Z = 1.96, the corresponding Z-score for the 95% CI

P = Proportion = 50%

W = Margin of error = 5% = 0.05

$$n=\frac{\left(1.96)2\;x\;0.5(1-0.5\right)}{(0.05)2}=384$$

By considering 10% non-response rate and a design effect of 1.5 the final sample size was 635. Finally, participants`households were accessed using a cluster sampling technique.

From 22 kebeles, 8 kebeles (Kebele 7, Kebele 8, Kebele 9, Kebele 13, Kebele 16, Kebele 17, Kebele 18, and Kebele 20) were selected by using the lottery method, then from each kebele one to two Ketena/s (the lowest administrative cluster) were selected depending on the number of households. The selected Ketena/s were considered as clusters and all households in the selected Ketena were included. Either of the parents in the household was interviewed or one family member age above 18 years was the respondent in the household whenever the parents were not available at the time of data collection.

### Operational definitions

#### Adherence towards COVID-19 mitigation measures

Was a composite variable generated from handwashing, using a facemask, keeping physical distance, not travel to a crowded place, homestay, and not travel to anyplace out of the city in the last 14 days. Hence, an individual was considered as having good adherence towards COVID-19 mitigation measures if he/she was able to answer ‘yes’ to the median and above of the aforementioned composite variables.

#### Information exposure

Respondents were asked whether they heard or not about the various aspects of COVID-19. The responses were coded as yes or no and those who responded with a median and above scores of the information exposure assessment questions were consideredas having a good information exposure level about COVID-19.

#### Good knowledge

Participants who responded with a median and above scores of the knowledge items about COVID-19 were labeled as having good knowledge otherwise poor knowledge.

#### Favorable attitude

Participants who responded with a median and above scores of the attitude questions about the COVID-19 and its preventive measures were labeled as having a favorable attitude otherwise unfavorable attitude.

#### Risk perception of COVID-19 infection

Risk perception was measured by two psychological dimensions; perceived susceptibility and perceived severity. The first dimension was proxied by how likely one considered oneself (his/her families) would be infected with COVID-19 if no preventive measure will be taken. The second dimension was proxied by how one rated the seriousness of symptoms caused by COVID-19, their perceived chance of having COVID-19 cured and that of survival if infected with COVID-19. By combining the two dimensions, five items with five response options were asked to determine the respondents’ levels of risk perception [23].

### Study variables

The outcome variable of this study was adherence towards COVID-19 mitigation measures, while others like socio-demographic, information exposure related characteristics, risk perception of COVID-19, knowledge about COVID-19, and its mitigation strategies, mode of transmissions, attitude towards COVID-19 and its prevention measures were the explanatory variables.

### Data collection tools and procedures

Data regarding the socio-demographic, information exposure, risk perception of COVID-19, and precaution measures adoption and community’s misconception about COVID-19 were collected through face-to-face interview using a structured questionnaire adapted from different literatures. Respondents were asked about the sources of information about COVID-19 and how much they trust those sources. They were also asked about the types of information that they wanted to receive. Participants were interviewed whether they performed precautionary measures including avoiding handshaking, adopting hand washing, and practicing physical distancing. Data were collected by BSc nurses and strictly followed by supervisors who managed the overall data collection process. A one-day training was given to the data collectors and supervisors about the purpose of the study, data collection tools, collection techniques, and ethical issues during the selection of the study participants and collection of the data. All responses to closed and open questions were written down manually by the interviewers. The supervisors assessed the consistency and completeness of data on a daily basis (S1 Table).

### Statistical analysis

The data entry was performed using the statistical program Epi-Data version 4.6 and then exported into STATA version 14 for analysis. Descriptive statistics was carried out and presented with narration and tabulation. Binary logistic regression (Bivariable and multivariable) was performed to identify statistically significant variables using a cut-off p-value < 0.2 in the bivariable analysis to identify candidate variables for multivariable logistic regression. Adjusted odds ratio with a 95% confidence interval was used to declare statistically significant variables on the basis of p-value <0.05 in the multivariable binary logistic regression model. Hosmer and Lemeshow goodness of fit test was performed and the decision was made at P>0.05.

### Quality assurance mechanisms

To assure the quality of the data, the tool was prepared first in English and then translated into the local language (Amharic) by language experts in English and Amharic languages. Data collectors and supervisors were trained on the data collection process for one day. A pretest was conducted from 5% of the total sample size in sub-city which is not selected for actual data collection. Appropriate modifications such as wording, changing terms, rephrasing for better understanding, deleting, and adding some information for clarity were made on the tool accordingly. Data collection was closely monitored by investigators and supervisors. Moreover, the data quality was assured by using statistical parameters for assessing the validity of the collected data.

Ethical clearance was obtained from the Institutional Review Board (IRB) of University of Gondar and an official permission letter was gained from the city administrative office. Written informed consent was obtained from each participant before conducting the actual data collection process. Any identifiable issues were eliminated to ensure confidentiality. Furthermore, appropriate infection prevention practices and principles related to COVID-19 were considered during the data collection process. Data collectors provided health education for the household after the interview has been completed based on the gaps identified as appropriate.

## Results

### Respondents’ sociodemographic characteristics

Of the overall sample required (N = 635), 623 participants were included in the study, giving a response rate of 98.1%. The mean (±SD) age of the respondents was 36.3 (= ±13.2) years, ranging from 18 to 80 years. Above a quarter of the respondents, 27.9% were in the age group of 34–45 years. Around two-thirds of the study participants were married (373, 59.87%) and 402 (64.5%) were females. Four hundred thirty-three (69.5%) were orthodox by religion. Regarding occupation, nearly three-fourth (448, 71.91%) of the participants were unemployed. Furthermore, on average, 4 and above people lived in the same household at the time of the study (SD = 2.04, min = 1, max = 14) (Table 1).

**Table 1:** Socio-demographic and personal characteristics of the study participants among Gondar City residents, Northwest, Ethiopia, 2020 (n = 623).

Variables	Frequency (n)	Percent (%)
Age (in years)		
18–26	163	26.2
27–33	150	24.1
34–45	174	27.9
>45	136	21.8
Sex		
Male	221	35.5
Female	402	64.5
Current marital status		
Unmarried	250	40.1
Married	373	59.9
Religion		
Orthodox	433	69.5
Muslim	154	24.7
Protestant	27	4.3
Others	9	1.5
Educational status		
No formal education	125	20.1
Primary education	101	16.2
Secondary education	195	31.3
College and above	202	32.4
Occupation		
Unemployed	448	72
Employed	175	28
Household size		
1–3	178	28.6
4–6	344	55.2
7 and above	101	16.2
Self-perceived health status		
Good	564	90.5
Bad	59	9.5
Perceived dangerousness of COVID-19		
Dangerous	570	91.5
Like the common cold/flu	53	8.5
Worry about COVID-19		
Worried	444	71.3
Not worried	109	17.5
Worried as it is common cold/flu	70	11.2

### Knowledge, attitude, risk perception, and information exposure related factors

Among all respondents, nearly half (49.3%) had poor knowledge about COVID-19 and only 57.5% and 52% of the respondents had a favorable attitude towards COVID-19 and its preventive measures, respectively. About 144 (23.11%) of the respondents had high risk perception of coronavirus. Furthermore, only 29.05% of the participants had good exposure to information about the various aspects of COVID-19. Of these, 84.75%, 84.59% and 43.18% of the respondents heard about COVID-19 symptoms, mode of transmission, and distribution of cases, respectively (Table 2).

**Table 2:** Knowledge, attitude, risk perception, and information exposure of the study participants about COVID-19 among Gondar City residents, Northwest, Ethiopia, 2020 (n = 623).

Variables	Frequency	Percent
**Knowledge about COVID-19**		
Poor knowledge	307	49.3
Good knowledge	316	50.7
**Attitude towards COVID-19**		
Unfavorable attitude	265	42.5
Favorable attitude	358	57.5
**Attitude towards prevention measures of COVID-19**		
Unfavorable attitude	229	48
Favorable attitude	324	52
**Risk perception of COVID-19**		
High risk	144	23.11
Low risk	479	76.89
**Heard about COVID -19 complications**		
Yes	144	18.30
No	509	81.70
**Heard about preventive measures taken by the government**		
Yes	248	39.81
No	375	60.19
**Heard about COVID -symptoms**		
Yes	528	84.75
No	95	15.25
**About COVID19 transmissions**		
Yes	527	84.59
No	96	15.41
**About distribution of COVID -19 cases**		
Yes	296	43.18
No	354	56.82
**Overall information exposure of the community**		
Good	181	29.05
Poor	442	70.95
**Correctly know COVID-19 symptoms**		
Correct	378	60.67
Incorrect	245	39.30
**Knows the COVID-19 mode of transmissions**		
Yes	361	57.94
No	262	42.05

### Adherence towards COVID-19 mitigation measures

The findings of this study indicated that nearly half of the study participants (**48.96% (95% CI: 45.05%, 52.89%))** had poor adherence towards COVID-19 mitigationmeasures. Among the mitigation strategies, hand washing was the commonest one practiced by the respondents (73.84%), while most (67.58%) of the participants failed to use a face mask (Table 3).

**Table 3:** Proportions of community’s adherence towards specific mitigation measures of COVID-19 among Gondar City residents.

Mitigation measures	Category	Proportion (95%CI)
Keeping physical distance 2 and above meters	Yes	55.06 (51.12, 58.93)
	No	44.94 (44.07, 48.88)
Use facemask when traveling out of home	Yes	32.42 (28.85, 36.21)
	No	67.58 (63.79, 71.15)
Travel to a crowed place	Yes	59.55 (55.63, 63.35)
	No	40.55 (36.65, 44.37)
Hand washing by soap and water in the past 2weeks	Yes	73.84 (70.23, 77.15)
	No	26.16 (22.85, 29.77)
Home stay	Yes	59.23 (55.31, 63.03)
	No	40.77 (36.96, 44.69)
Travel history in the past 2 weeks	Yes	15.41 (12.78, 18.47)
	No	84.59 (81.53, 87.22)
Overall adherence towards COVID_19 mitigation measures	Poor	48.96 (45.05, 52.89).
	Good	51.04 (47.11, 54.96)

Adherence towards COVID-19 mitigation measures was a composite variable generated from handwashing, using a facemask, keeping physical distance, not travel to a crowded place, homestay, and not travel to anyplace out of the city in the last 14 days. Hence, an individual was considered as having good adherence towards COVID-19 mitigation measures if he/she was able to answer ‘yes’ to the median and above of the aforementioned composite variables.

### Factors associated with adherence towards COVID-19 mitigation measures

The association between all potential independent variables and adherence towards COVID-19 mitigation measures were analyzed using binary logistic regression. Accordingly, on bivariable binary logistic regression analysis, predictor variables such as sex, household size, level of information exposure, self-perceived health status, perceived dangerousness, knowledge about COVID-19, attitude towards COVID-19 preventive measures, correctly know COVID-19 symptoms, knows the COVID-19 mode of transmissions, risk perception of COVID-19 were explored to significantly influenced the adherence of the community towards mitigation measures against COVID-19. After controlling for confounders in a multivariable binary logistic regression analysis, sex, level of information exposure, attitude towards COVID-19 preventive measures, and risk perception of COVID-19 remained to significantly influence the adherence of the community towards COVID-19 mitigation measures.

Hence, female respondents had 2.39 times better adherence than males towards COVID-19 mitigationmeasures [AOR: 2.39; 95%CI (1.66, 3.45)]. Respondents that had a good level of information exposure about COVID-19 were 1.58 times more likely to have good adherence towards COVID-19 mitigation measures than their counterparts [AOR: 1.58; 95%CI (1.03, 2.43)]. And also, study participants who had favorable attitude towards COVID-19 preventive measures were 2.54 times more likely to adhere towards the mitigationmeasures against COVID-19 than respondents who had an unfavorable attitude towards COVID-19 preventive measures [AOR: 2.54; 95%CI (1.79,3.60)]. Furthermore, respondents who had high risk perception of COVID-19 were 39% less likely to have good adherence towards mitigation measures against COVID-19 than their counterparts [AOR: 0.61; 95% CI (0.41, 0.92)] (Table 4).

**Table 4:** Factors associated with adherence towards COVID-19 mitigation measures among Gondar City residents.

Variable name	Category	Frequency	COR (95%CI)	AOR(95%CI)	P_value
Sex	Male	221	1	1	
	Female	402	2.02(1.45, 2.82)	2.39(1.66, 3.45)**	**0.001**
Household size	1–3	178	1	1	
	4–6	344	1.89(0.82, 1.70)	0.98(0.66,1.45)	0.90
	7 and above	101	1.67(1.02,2.75)	1.33(0.77, 2.29)	0.31
Self-perceived health status	Good	564	1	1	
	Bad	59	0.63(0.37, 1.09)	0.96(0.53, 1.75)	0.91
Perceived dangerousness	Dangerous	570	2.16(1.19, 3.90)	1.64(0.86, 3.11)	0.31
	Like the common cold/flu	53	1	1	
Level of information exposure	Good	181	2.27(1.58, 3.24)	1.58(1.03, 2.43)*	**0.04**
	Poor	442	1	1	
Knowledge about COVID-19	Poor knowledge	307	0.41(0.30, 0.57)	0.79(0.46, 1.34)	0.38
	Good knowledge	316	1	1	
Attitude towards COVID-19 preventive measures	Unfavorable attitude	229	1	1	
	Favorable attitude	324	2.68(1.94,3.71)	2.54(1.79,3.60)**	**0.001**
Correctly know COVID-19 symptom	Correct	378	1	1	
	Incorrect	245	0.44 (0.32, 0.61)	0.75 (0.45, 1.24)	0.26
Knows the COVID-19 mode of transmission	Yes	361	1	1	
	No	262	0.41 (0.30, 0.58)	0.76(0.48, 1.19)	0.23
Risk perception of COVID-19	High risk	144	0.57(0.39,0.83)	0.61 (0.41, 0.92)*	**0.02**
	Low risk	479	1	1	

*shows significant at p<0.05;

**implies significant at P<0.001

Hosmer and Lemeshow the goodness of fit test P = 0.134

## Discussion

Since the emergence of COVID-19 pandemic, there is no definitive treatment found. Therefore, the best alternative to control the spread of this pandemic is adherence towardsthe recommended mitigation startegies. This study assessed the adherence of the residents of Gondar city towards COVID-19 mitigation measures since the beginning of the outbreak in Ethiopia in March 13, 2020.

Accordingly, the study revealed that the overall adherence of the communitytowards COVID-19 mitigation measures was 51.01%. Of the specific mitigation measures, 73.84% of the respondents reported that they had been frequently washing their hands with water and soap, which is comparable with the two studies conducted in Jimma, Ethiopia (76%) [24] and (77.3%) [21]. However, the result of our study is lower than studies carried out in China (79.44%) [25], Kansans, USA, (97%) [26], Egypt (87.6%) [27], and Malaysia (87.8%) [28]. The possible explanation may be due to the differences in the study population, socio-demographic characteristics and the measurement tools used across the studies. For instance, when we compare our study participants with that of China, our study was conducted on a community whereas the study conducted in China was on healthcare workers whom would have better prior knowledge and experience about mitigationmeasures of COVID-19 than our study participants. Additionally, the study participants of the study conducted in China had taken education about hand hygiene and other infection control measures [25]. As a result, the healthcare workers who have prior knowledge and experience as well as the training might increase their adherence towards mitigation measures against COVID-19. Furthermore, there is intermittent water supply in most parts of Ethiopia and limited hand washing facilities which in turn negatively affected the adherence of the community towards hand hygiene in our study.

The other specific mitigation measures were no travel to crowded places and staying at home. As such, this study noted that 40.55% of the respondents reported that they hadn’t traveled to crowded places that means they had good adherence towards the principle of avoiding traveling to crowded places so as to prevent the spread of the pandemic. This finding is higher than a study conducted in Jimma (33.2%) [21]. Nevertheless, this finding is lower than studies done in Egypt (87.1%) [27] and Malaysia (83.4%) [28]. Regarding staying at home, 59.23% of the respondents reported that they stayed at home. This finding is lower than a study conducted in Egypt (96.1%) [27]. The possible explanation for the difference might be the living conditions in our study setting, there is mostly high social and physical interaction leading to overcrowding. There are also frequent religious activities in Gondar which forced the respondents to go to religious places. Similarly, unemployment is common in the country, so most people will go to crowded places, for they need to make money and satisfy their basic needs. Moreover, the infection emerged earlier in Egypt than Ethiopia which forced the Egyptians to stay at home and avoid traveling to crowded places. Hence, our study participants were negatively influenced by the above conditions about the adherence of not traveling to crowded places and staying at home.

This study found out that the adherence of the community towards wearing a facemask as a mitigation measure was the least commonly used methods of mitigating the spread of COVID-19 infection in the study area. In this regard, 67.58% of the study participants didn’t use a face mask while going out of their home which is higher than studies conducted in USA (23%) [26] and Egypt (43%) [27]. The possible reasons could be most of the residents might not afford facemasks in order to use them on a daily basis when compared to residents of USA and Egypt.

This study identified that sex, level of information exposure, attitude towards COVID-19 preventive measures and risk perception of COVID-19 had statistically significant association with good adherence towards COVID-19 mitigation measures. Accordingly, female respondents were 2.39 times more likely to have good adherence towards the mitigation measures of COVID-19. This finding is in line with studies conducted in the Netherlands [29], Cyprus [30], and United States [31]. The possible justification might be the majority of males work outside their home by moving from one place to another place. As a result, mitigation measures might not be available and suitable for each place. In addition to this, because males move from place to place more often, they use transportation services, which will be difficult to comply with physical distancing. On the other hand, in our context, females bear a huge burden of childcare, so they may fear transmitting the disease to their children if they didn’t adhere towards the proper mitigation measures. Therefore, females might implement greater adherence towards mitigation measures of COVID-19.

This study showed that the respondents whohad a good level of information exposure were 1.58 times more likely to have good adherence towards COVID-19 mitigation measures than their counterparts. This finding is congruent with a study conducted in the Netherlands [29] which revealed that low information seeking behavior was inversely associated with compliance. This might be due to the fact that if the population had prior information about the utilization and advantage of the mitigation measures, they might develop a good attitude towards these preventive measures which in turn increase theiradherence.

The other significant factor affecting the adherence of the community towards COVID-19 mitigation measures in this study was attitude towards COVID-19 preventive measures. In this regard, the respondents who had a favorable attitude towards COVID-19 preventive measures were 2.54 times more likely to adhere towardsthe mitigation measures than respondents who had an unfavorable attitude towards COVID-19 preventive measures. This result is in agreement with a study carried out in Jimma, Ethiopia [24]. The possible explanation might be that the respondents who had a favorable attitude towards COVID-19 preventive measures might trust the science of mitigation measures and comply with the instructions of these guidelines.

Lastly, respondents who had a high risk perception of COVID-19 were 39% less likely to have good adherence towards COVID-19 mitigation measures than their counterparts. The plausible explanation might be due to the link between the high risk perception of COVID-19 and anxiety. As a result, this anxiety might lead to unnecessary behaviors associated with an increased level of impairment within the individual and the community at large [32]. Thus, the community’s adherence towards mitigation measures would be negatively affected by high risk perception of COVID-19. This finding is in contrast with a study conducted in United States [33] which revealed that as individual’s perception of risk increases, they highly engage in risk prevention behaviors. Additionally, this finding is also in contrast with a study done in United Kingdom [34] and Slovenia [35] which showed that desensitization to risk or genuine reductions in risk might lead to reduction in mitigation measures utilization.

## Limitations of the study

This study acknowledged some important possible limitations that should be considered when interpreting the results. First, the study was cross-sectional, a design that does not permit establishing cause-effect relationships. Second, social desirability bias might be introduced.

## Strength of the study

Through this community based survey, it was possible to conduct a face-to-face interview and observation with maximum precaution than a simple telephone survey to evaluate the real response and adherence of the community towards mitigation measures against the pandemic despite the lockdown effect where many people were confined at home.

## Conclusions

Our findings have indicated that nearly half of the study participants had poor adherence towards COVID-19 mitigation measures. Sex, level of information exposure, attitude towards COVID-19 preventive measures, and risk perception of COVID-19 were factors, which significantly influenced the adherence of the community towards COVID-19 mitigation measures. Therefore, it is crucial to track adherence responses to the COVID19 measures, scale up the community’s awareness of COVID-19 prevention and mitigation strategies through appropriate information outlets such as mainstream media on prevention strategies of COVID-19, and rely on updating information from TV, radio, and healthcare workers about COVID-19.

## Supporting information

S1 Table English version questionnaire. (DOCX)

S1 Dataset (XLS)

## Abbreviations

AOR: Adjusted Odds Ratio
CI: Confidence Interval
COR: Crude Odds Ratio
COVID-19: Coronavirus disease 19
MERS: Middle East Respiratory Syndrome
OR: Odds Ratio
SARS: Severe Acute Respiratory Syndrome
SD: Standard Deviation
SPSS: Statistical Package for Social Sciences
TV: Television
WHO: World Health Organization
